The article "Role of microRNA-130a in the pathogeneses of obstructive sleep apnea hypopnea syndrome-associated pulmonary hypertension by targeting the GAX gene" was retracted in 2021. Reasons: errors in the methods; errors in the results or conclusions.

# Role of microRNA-130a in the pathogeneses of obstructive sleep apnea hypopnea syndrome-associated pulmonary hypertension by targeting the *GAX* gene

**DOI:** 10.1097/MD.0000000000006746

**Published:** 2017-05-19

**Authors:** Zhe An, Dan Wang, Guang Yang, Wen-Qi Zhang, Jin Ren, Jin-Ling Fu

**Affiliations:** a Department of Cardiology, China-Japan Union Hospital of Jilin University; b Department of Breast Surgery, The Second Hospital of Jilin University; c Department of Molecular Biology, College of Basic Medical Sciences, Jilin University; d Department of Respiratory Medicine, the Second Hospital of Jilin University; e Department of Ophthalmology, The Second Hospital of Jilin University, Changchun, Jilin, P.R. China.

**Keywords:** *GAX* gene, MicroRNA-130a, obstructive sleep apnea hypopnea syndrome, pathogenesis, pulmonary hypertension

## Abstract

**Objective:**

The purpose of this study was to elucidate the role of microRNA-130a (miR-130a) in obstructive sleep apnea hypopnea syndrome (OSAHS)-associated pulmonary hypertension (PHT) by targeting the growth arrest-specific homeobox (*GAX*) gene.

**Methods:**

A total of 108 patients with OSAHS-associated PHT were recruited as the OSAHS-associated PHT group and 110 healthy individuals were randomly selected as the normal control group. Human umbilical vein endothelial cells (HUVECs) were selected and divided into the control, miR-130a mimic, mimic negative control (NC), miR-130a inhibitor, and inhibitor-NC groups. The dual luciferase reporter gene assay was used to identify the relationship between miR-130a and the *GAX* gene. The quantitative real-time polymerase chain reaction (qRT-PCR) and Western blotting were applied for the relative expressions of miR-130a and the mRNA and protein expressions of *GAX*. Serum levels of endothelin-1 (ET-1), vascular endothelial growth factor (VEGF), nitric oxide (NO), and super oxide dismutase (SOD) were detected. Cell apoptosis and angiogenic activity were analyzed by flow cytometry and cell tube formation assay.

**Results:**

*GAX* was a target gene of miR-130a. Compared with the normal control group, the relative expression of miR-130a and the serum levels of ET-1 and VEGF were increased, whereas the mRNA expression of *GAX* and the serum levels of NO and SOD were decreased in the OSAHS-associated PHT group. Compared with the control, mimic-NC, and inhibitor-NC groups, the relative expressions of miR-130a in the miR-130a mimic group were enhanced, whereas the expression of miR-130a in the miR-130a inhibitor group was reduced. However, the mRNA and protein expressions of *GAX* showed an opposite trend in the miR-130a mimic and miR-130a inhibitor groups. In comparison to the control, mimic-NC, and inhibitor-NC groups, the miR-130a mimic group had an increase of ET-1 and VEGF expressions, whereas the expressions of NO and SOD were reduced. However, the miR-130a inhibitor group exhibited an opposite trend. The apoptosis rate and tube formation number in the miR-130a mimic group were obviously increased, whereas the miR-130a inhibitor group showed an obvious decrease.

**Conclusion:**

These data provided strong evidence that miR-130a may be involved in the progression of OSAHS-associated PHT by down-regulating *GAX* gene.

## 1 Introduction

Obstructive sleep apnea hypopnea syndrome (OSAHS) is a common clinical condition defined by excessive daytime sleepiness (EDS), loud snoring, and witnessed breathing pauses and is belong to sleep-disordered breathing (SDB).^[1–4]^ The main clinical manifestations included persistent loud snoring and fatigue or excessive daytime sleepiness.^[5–8]^ Old people reported a history of OSAHS more frequently than middle-aged people (30% and 80% vs 2%–4%), and studies have strongly shown that OSAHS has also been related to chronic diseases and might have a dysfunction of the arousal system control.^[1,9–11]^ The symptoms of OSAHS may include reduced sleep quality because of abnormal position during sleep, decreased life quality because of mood disorders, and cognitive problems at all ages.^[12,13]^ Fein et al^[14]^ showed that pulmonary hypertension (PHT) had a close relationship with chronic obstructive lung disease (COPD) and sleep-disordered breathing. PHT is a pathologic lung condition that occurs owing to vascular remodeling, invoking an increase in right ventricular afterload which causes right ventricular hypertrophy, right heart failure, and ultimately death.^[15]^ EDS is one of symptoms of OSAHS, and the accumulated evidence indicates a close association between EDS and an increased risk of hypertension.^[16]^

MicroRNAs (miRNAs) can monitor the expression of gene by 2 ways, which decided by the degree of complementarity with the mRNA targets, to restrain translation or induce mRNA degradation, and some miRNAs are able to regulate immune and neuronal processes.^[17,18]^ Many genes related to different cancer pathways have been implicated in miR-130a expression, such as growth arrest-specific homeobox (*GAX*).^[19]^ Recently, it has been found that miRNA-130a plays an important role in different diseases of human, such as hepatocellular carcinoma, ventricular arrhythmias, hepatic insulin sensitivity and liver steatosis, endothelial progenitor cell dysfunction and human colorectal cancer.^[20]^ The *GAX* gene, also called MEOX2, a part of homeobox gene family, encodes a homeodomain-containing transcription factor and the expression of *GAX* exists both in vascular smooth muscle cells (VSMCs) and vascular endothelial cells (ECs).^[21]^ A transcription factor encoded by *GAX* gene can regulate proliferation, differentiation, and migration in different cell types, meanwhile, *GAX* gene may play a part in hypoxia-induced PHT by modulating the proliferation of pulmonary artery smooth muscle cells (PASMCs).^[22]^

miRNAs in human PHT as an important role in the diagnosis of PHT has been identified by many studies, previous study has validated that the *GAX* gene play a part in hypoxia-induced PHT through regulating the proliferation of VSMCs. Bertero et al^[23]^ demonstrated that miR-130a has a positive influence in promoting vascular extracellular matrix (ECM) remodeling in PHT. The evidence also showed that the *GAX* gene was a key point in VSMCs proliferation and migration.^[24]^ Moreover, PHT is defined by pulmonary arteriolar remodeling with massive pulmonary VSMC proliferation.^[25]^ However, the correlations among miRNAs, *GAX* gene, and OSAHS-associated PHT have not been reported yet. Therefore, this study was performed to explore the effect of miR-130a on OSAHS-associated PHT by targeting the *GAX* gene.

## 2 Subjects and methods

### 2.1 Subjects

Between October 2013 and April 2016, a total of 108 patients (68 males, 40 females, mean age: 54.65 ± 7.81 years) with OSAHS-associated PHT were selected as the OSAHS-associated PHT group from the Second Hospital of Jilin University. The inclusion criteria were as follows: (1) patients who were diagnosed as OSAHS according to Guidelines for the diagnosis and treatment of obstructive sleep apnea hypopnea syndrome (2011), and pulmonary hypertension (PHT) was defined as mean pulmonary arterial pressure (mPAP) ≥ 25 mm Hg.^[26]^ (2) Patients without bronchial asthma, active pulmonary tuberculosis, lung cancer, primary bronchial dilation, pneumoconiosis, and other lung restrictive ventilatory dysfunction; (3) patients without other serious system diseases of cardiovascular, nerve, endocrine, blood system, liver, kidney, and malignant tumor. The exclusion criteria were as follows: (1) patients who are unwilling to cooperate or unable to communicate. (2) Patients with incomplete clinicopathological data. Meanwhile, 110 healthy subjects (57 males, 53 females; mean age: 53.28 ± 7.26 years) were randomly selected as the normal control group. The blood of patients with OSAHS-associated PHT and healthy subjects were preserved in cryogenic vials. Informed consents were obtained from all study subjects and/or their legal guardians. This study complied with the guidelines and principles of the ethics committee on clinical trials of the Second Hospital of Jilin University.

### 2.2 Cell culture and transfection

Human umbilical vein endothelial cells (HUVECs) were purchased from ATCC (American type culture collection, Rockville, MD), which were maintained in RPMI-1640 medium (Hyclone, Utah) in the presence of 10% inactivated fetal bovine serum (FBS, Gibco), streptomycin (100 mg/mL, Hyclone, Utah), and penicillin (100 U/mL, Hyclone, Utah) at 37°C with 5% CO_2_ in an incubator (Thermo Fisher Scientific, MA). HUVECs were spread on the plate before transfection and conventionally incubated for 24 hours, and then refreshed with 2 mL RPMI-1640 medium 1 hour before transfection. Transfection mixture was configured according to the manufacturer's guidelines of Lipofectamine 2000 kit (Invitrogen Corporation, Carlsbad, CA). The cells were divided into 5 groups: the Control (without any plasmid transfection), miR-130a mimic, mimic negative control (NC), miR-130a inhibitor and inhibitor-NC groups. Transfection mixture was added and incubated at 37°C after the RPMI-1640 medium was sucked out from each well. All the successfully transfected cells were identified before the biological assay.

### 2.3 Oligonucleotide synthesis and vector construction

The oligonucleotide sequences of the miR-130a mimic, mimic-NC, miR-130a inhibitor, and inhibitor-NC groups were shown in Table 1, which synthesized by Shanghai Ji Ma company (Shanghai, China). To test the relationship between miR-130a and the *GAX* gene, a *GAX* 3′-Untranslated region (UTR) fragment containing the miR-130a binding sites in the 3′-UTR of the human was amplified and implanted into the psiCHECK2 vector (Promega Corporation, Madison, WI), constructing the plasmid of psiCHECK2-*GAX*-3′- UTR-wild type (*GAX* wild) for the expression of miR-130a and *GAX* binding sites and the plasmid of psiCHECK2-*GAX*-3′- UTR-mutant (*GAX* mutant) for expressing miR-130a and *GAX* non-binding site, as a spare after sequencing.

**Table 1:** The sequences of oligonucleotides and vector construction.

### 2.4 Dual luciferase reporter gene assay

HUVECs were seeded in 96-well plates at a density of 4 × 10^4^ cells per well 24 hours and then refreshed with RPMI-1640 medium 1 hour before transfection. Cells were incubated with transfection mixture which was configured by the manufacturer's guidelines of Lipofectamine 2000 (Invitrogen Corporation, Carlsbad, CA) kit for 24 hours at 37°C. Transcriptional activity was evaluated using the dual luciferase reporter gene assay system (Promega Corporation, Madison, WI). The co-transfection groups were the control (without any plasmid transfection), miR-130a mimic, mimic-NC, miR-130a inhibitor and inhibitor-NC groups. All the successfully transfected cells were identified before the biological assay.

### 2.5 Quantitative real-time polymerase chain reaction (qRT-PCR)

The miRNA was extracted according to the manufacturer's guidelines of miRNeasy Mini kit (Qiagen). RNA of HASMCs was extracted using TRIzol reagent (Invitrogen) and the RNA concentration was detected by NanoDrop2000 (Thermo), then reserved at –80°C. And qRT-PCR was performed with the gene sequence published in the Genbank database using the Primer 5.0 software. The primers as shown in Table 2 were synthesized by Shanghai Ji Ma company (Shanghai, China). miRNA was subjected to reverse transcription using One Step PrimeScript miRNA cDNA Synthesis Kit (Perfect Real Time) (Takara), and the condition was at 37°C for 1 hour (poly (A) tailing and reverse transcription), heat shock was performed at 85°C for 5 seconds (enzyme inactivation reaction). The RT-PCR conditions of miRNA were as follows: 42°C for 5 minutes and 95°C for 10 seconds, followed by 40 cycles at 95°C for 5 seconds, 60°C for 1 minute and 72°C for 15 seconds. The non-miRNA RT-PCR reaction system was conducted according to the manufacturer's guidelines of One Step SYBR PrimeScript PLUS RT- PCR Kit (Takara), the PCR conditions were 40 cycles of 42°C for 5 minutes, 95°C for 10 seconds, 94°C for 5 seconds, 58°C for 30 seconds, and 72°C for 15 seconds. U6/β-actin was used as an internal reference, and the reliability of PCR results was determined using dissolution curve and analyzed by the DCT method: ΔCT = Ct (target gene) – Ct (reference gene), ΔΔCt = ΔCt (experimental group) – ΔCt (control group). miRNA expression of target genes was determined by 2^-^ΔΔ^Ct^ methodology.^[27]^

**Table 2:** Primer sequences of microRNA and signaling pathway-related genes.

### 2.6 Western blotting

Concentrations of protein were determined by BCA kit (Boster Co., Ltd., Wuhan, China). The extracted protein was diluted in the sample buffer and boiled at 95°C for 10 minutes, and the sample was loaded into 96-well plates (50 μg per well). Protein samples were separated by electrophoresis in 10% polyacrylamide (Boster Co., Ltd., Wuhan, China), followed by wet transfer process utilizing the polyvinylidene fluoride (PVDF) membrane with voltage electrophoresis of 80 V to 120 V and transfer of 100 MV voltage for 70 minutes. Membranes were blocked in 5% bovine serum albumin (BSA) for 1 hour at room temperature, and then incubated overnight at 4°C with diluted primary antibodies *GAX* and β-actin (both 1:500 dilution, Abcam). After being washed with TBST 3 times for 5 minutes each time, the membranes were incubated with diluted second antibodies (1:1000 dilutions, Abcam) at room temperature for 1 hour, and washed 3 times with BSA for 5 minutes. The samples were then developed using chemical luminescence reagent (ECL). Meanwhile, β-actin as a reference standard and bands were visualized using the Gel Doc EZ Imager (Bio-rad, CA). The gray values of the target bands were analyzed by the Image J software.

### 2.7 Detection of cytokines in serum

Endothelin (ET) Kit was provided by the East Asia Institute of Immune Technique, General Hospital of Chinese PLA. The samples (1 mL) were transferred to a centrifuge tube containing 10% Na2EDTA (15 μL) and aprotinin (20 μL), centrifuged at 3000 rpm for 10 minutes at 4°C and the plasma was isolated. The reaction solution was configured by the operating manual of kit, then mixed, incubated at room temperature for 15 minutes and centrifuged at 3500 rpm for 20 minutes, and then the supernatant was abandoned. ^125^I-ET (radioactive iodine) and standard products/samples were combined with ET-1 antibody simultaneously and competitively. The concentration of ET was discovered from the radioactivity content by reference to standard curves. Samples (1 mL) were mixed with 0.5 mL of 0.02% 4-hydroxy (solubilized in dimethylformamide, 2 mol/L HCl = 1:1, Sigma-Aldrich, St. Louis, MO), and incubated on ice for 5 minutes. Samples were added with 50 μL of 8% Na_2_S_2_O_3_ (Sigma-Aldrich, St. Louis, MO) and placed at room temperature for 10 minutes, then added with 1.5 mol/L NaOH (Sigma-Aldrich, St. Louis, MO) (0.5 mL) and placed at room temperature for 10 minutes. The relative fluorescence intensity was measured with the thermo fluorescence spectrophotometer and curves were made by using NaNO_2_ (Sigma-Aldrich, St. Louis, MO) as internal standard, and then the relative concentration of nitric oxide (NO) was calculated. The test was operated according to the manufacturer's instructions of VEGF ELISA Kit (Roche, Mannheim, Germany). ELISA kit was placed at room temperature for 20 minutes when the washing liquid, standard sample, and reaction system were prepared. The optical density (OD) value (450 nm) of each well was detected by the microplate reader (BioTek Synergy 2) in 3 minutes after termination of the reaction. The standard curve was drawn by the OD value and the value of vascular endothelial growth factor (VEGF) was detected. Super oxide dismutase (SOD) Kit was provided by Nanjing Jiancheng Bioengineering Institute (Jiangsu, China) and the reaction solution was configured by the manufacturer's instructions of kit, and then incubated at room temperature for 10 minutes after mixed. Absorbance at 550 nm was measured by using a spectrophotometer (type 722, Thermo), SOD activity (U/mL) = (control tube OD – evaluated tube OD)/control tube OD/50%.

### 2.8 Flow cytometry

After 24 hours of transfection, the HUVECs were digested by trypsin and collected by centrifugation. After centrifugation, cells were washed with cold phosphate buffered saline (PBS) and suspended at a final concentration of 1 × l0^6^ cells/mL in PBS-containing calcium. The 100 μL of cell suspension was transferred into a test tube at room temperature, mixed with propidium iodide (10 mg/mL) and RNase A (10 mg/mL), then incubated at 4°C for 30 minutes. Subsequently, 400 μL staining buffer was added into the cell suspension, and the apoptotic cells were detected by flow cytometry (BD Bioscience, Oxford, UK). And 10^4^ cells were analyzed using the Cell Quest software (Becton Dickinson) each time. Annexin V-positive cells were regarded as apoptotic cells, PI positive, and Annexin V-negative cells were necrotic cells. Furthermore, cells in the left upper quadrant were necrotic cells, and those in the left lower quadrant were normal cells; however, cells in the right upper quadrant were late apoptotic cells and those in the right lower quadrant were early apoptotic cells.

### 2.9 Tube formation assay

Pre-liquefied Matrigel (BD Company) (60 μL) was plated in sterilized 96-well plates (Corning, NY) and distributed evenly, and then incubated for 30 min at 37°C. The coagulated Matrigel was removed and cells in the logarithmic growth phase with a density of 1 × 10^5^ cells/mL were added into each well, and then cultured at 37°C with 5% CO_2_. After 24 hours, tube formation of cells in vitro was observed under a phase contrast microscope (Olympus, Tokyo Japan), and the number of branch points was quantitated at low magnification (100×) and photographed for observation at high magnification (400×).

### 2.10 Statistical analysis

Data were analyzed applying the statistical package for the social sciences (SPSS) version 21.0 (SPSS Inc.; Chicago, IL). Continuous data were displayed as (mean ± standard deviation), in which the differences between 2 groups were analyzed by the *t*-test and among multiple groups by 1-way analysis of variance (ANOVA). Categorical data were expressed as the ratio and percentage, and the differences among groups were compared by the chi-square test. Pearson correlation analysis was used to compare the correlation between the 2 variables. *P* < .05 indicated statistically significant.

## 3 Results

### 3.1 The target relationship between miR-130a and the GAX gene

The results of dual luciferase reporter gene assay indicated that compared with the control group, the transcriptional activity of *GAX* gene exhibited no remarkable difference in the mimic-NC and inhibitor-NC groups (*P* > .05). Only in *GAX* wild, in comparison to the control group, the transcriptional activity of *GAX* in the miR-130a mimic group was significantly decreased, whereas that in the miR-130a inhibitor group was notable increased (all *P* < .05) (Fig. 1).

**Figure 1:** The target relationship between miR-130a and *GAX* gene. Note: (A) two binding sites of miR-130a in *GAX* 3′-UTR; (B) miR-130a regulated *GAX* gene transcriptional activity by the dual luciferase reporter gene assay. *GAX* = growth arrest-specific homeobox gene, miR-130a = microRNA-130a.

### 3.2 Relative expressions of miR-130a and the mRNA expressions of GAX in serum of the OSAHS-associated PHT and control groups

The results of qRT-PCR indicated that compared with the normal control group, the mRNA expression of miR-130a was significantly increased in the OSAHS-associated PHT group, whereas the mRNA expressions of *GAX* was obviously decreased (all *P* < .05) (Fig. 2).

**Figure 2:** The relative expressions of miR-130a (A) and the mRNA expressions of *GAX* (B) in serum of the OSAHS-associated PHT and normal control groups using qRT-PCR. Note: ^∗^ = *P* < .05, *GAX* = growth arrest-specific homeobox gene, miR-130a = microRNA-130a, OSAHS = obstructive sleep apnea hypopnea syndrome, PHT = pulmonary hypertension, qRT-PCR = quantitative real-time polymerase chain reaction.

### 3.3 Serum levels of VEGF, ET, NO, and SOD in the OSAHS-associated PHT and control groups

The results of detection of the expression of cytokines (VEGF, ET, NO, and SOD) showed that compared with the normal control group, the expressions of ET-1 and VEGF were increased, whereas the expressions of NO and SOD were decreased in the OSAHS-associated PHT group (all *P* < .05) (Table 3).

**Table 3:** Serum levels of VEGF, ET, NO, and SOD in the OSAHS-associated PHT and normal control groups.

### 3.4 Relative expressions of miR-130a and the mRNA and protein expressions of GAX in 5 groups

The results of qRT-PCR and Western blotting revealed that the miR-130a expression and the mRNA and protein expressions of GAX exhibited no remarkable difference among the control, mimic-NC, and inhibitor-NC groups (all *P* > .05). Compared with the control group, the expression of miR-130a in the miR-130a mimic group was increased and that in the miR-130a inhibitor group was significantly reduced (all *P* < .05), whereas the mRNA and protein expressions of GAX exhibited an opposite trend (Fig. 3A and B). Pearson correlation analysis showed that the *GAX* gene was negatively correlated with miR-130a (*r* = –0.656, *P* < .05) (Fig. 3C).

**Figure 3:** The relative miR-130a expressions (A) and the mRNA (A) and protein expressions (B) of *GAX* in 5 groups. Note: (C) *Pearson correlation analysis* used to examine the *correlation between* the *GAX* gene and miR-130a. ^∗^ = *P* < .05 when compared with the control group, ^#^ = *P* < .05 when compared with the mimic-NC group, ^&^ = *P* < .05 when compared with the inhibitor-NC group, *GAX* = growth arrest-specific homeobox gene, miR-130a = microRNA-130a, qRT-PCR = quantitative real-time polymerase chain reaction, NC = negative control.

### 3.5 Serum levels of ET-1, NO, VEGF, and SOD in HUVECs in 5 groups

The levels of cytokines (ET-1, NO, VEGF, and SOD) validated that there was no difference among the mimic-NC and inhibitor-NC groups compared with the control group (*P* > .05). In comparison to the control and mimic-NC groups, the serum levels of ET-1 and VEGF were remarkably enhanced in the miR-130a mimic group, whereas the serum NO and SOD levels were remarkably reduced (all *P* < .05). Furthermore, compared with the control and inhibitor-NC groups, the serum levels of ET-1 and VEGF were remarkably decreased in the miR-130a inhibitor group, whereas the levels of NO and SOD were remarkably increased (all *P* < .05) (Table 4).

**Table 4:** The serum levels of ET-1, VEGF, NO, and SOD in HUVECs in 5 groups.

### 3.6 Correlations of the relative expressions of miR-130a, GAX and the serum levels of cytokines (ET-1, NO, VEGF, and SOD) in 5 groups

The results of Pearson correlation analysis indicated that the expressions of ET-1 and VEGF were positively correlated with the expression of miR-130a (*r* = 0.719, *r* = 0.802, respectively), whereas the serum levels of NO and SOD were negatively correlated with the miR-130a expression (*r* = –0.729, *r* = –0.843, respectively). There was a negative correlation in the expressions between ET-1, VEGF, and *GAX* (*r* = –0.795, *r* = –0.869, respectively); however, a positive correlation was shown in the comparison among the serum levels of NO and SOD and the mRNA expressions of *GAX* (*r* = 0.702, *r* = 0.855, respectively) (Fig. 4).

**Figure 4:** *Correlations* of the relative expressions of miR-130a, mRNA expressions of *GAX*, and serum levels of cytokines (ET-1, NO, VEGF, and SOD) in 5 groups by Pearson correlation analysis. Note: ET = endothelin, *GAX* = growth arrest-specific homeobox gene, miR-130a = microRNA-130a, NO = nitric oxide, VEGF = vascular endothelial growth factor, SOD = super oxide dismutase.

### 3.7 Cell apoptosis of HUVECs in 5 groups after transfection

The results of flow cytometry revealed that, compared with the control group, there was no statistically significant difference in the cell apoptosis rates of the mimic-NC and inhibitor-NC groups (*P* > .05); However, compared with the control and mimic-NC groups, respectively, the miR-130a mimic group had raised rate of cell apoptosis (*P* < .05). In the comparison of the control and inhibitor-NC groups, the miR-130a inhibitor group had reduced the cell apoptosis rate (both *P* < .05) (Fig. 5).

**Figure 5:** Cell apoptosis of HUVECs in 5 groups after transfection using flow cytometry. Note: ^#^ = *P* < .05 when compared with the mimic-NC group, ^&^ = *P* < .05 when compared with the inhibitor-NC group, HUVECs = human umbilical vein endothelial cells, miR-130a = microRNA-130a, NC = negative control.

### 3.8 The tube formation of HUVECs in 5 groups after transfection

The HUVECs tube formation assay founded that the tube formation exhibited no remarkable difference among the control, mimic-NC, and inhibitor-NC groups (the average number of branch points were 22, 24, and 20, respectively) (*P* > .05). Compared with the control and mimic-NC groups, tube formation in the miR-130a mimic group was obviously increased (mean value, 38) (*P* < .05). However, compared with the control and inhibitor-NC groups, the tube formation in the miR-130a inhibitor group was obviously decreased (mean value, 14) (*P* < .05) (Fig. 6). The results indicated that miR-130a promoted angiogenesis inhibited by the *GAX* gene.

**Figure 6:** The tube formation of HUVECs in 5 groups after transfection under the phase contrast microscope (400×). Note: ^∗^ = *P* < .05 when compared with the control group, ^#^ = *P* < .05 when compared with the mimic-NC group, ^&^ = *P* < .05 when compared with the inhibitor-NC group, HUVECs = human umbilical vein endothelial cells, miR-130a = microRNA-130a,NC = negative control.

## 4 Discussion

Evidence showed that the main clinical characteristic of OSAHS is defined by the disturbances in sleep structure and nocturnal hypoxemia and hypercapnia, which may lead to excessive sleepiness in the daytime, cardio-cerebrovascular events, and multiple organ injury that may gravely affect the quality of life (QOL).^[28]^ And PHT is defined by an imbalance with an increase in pulmonary vascular resistance and pulmonary artery pressures.^[29]^ This study explored the effect of miR-130a in OSAHS-associated PHT by targeting the *GAX* gene, our findings validate that miR-130a might limited the expression of *GAX* and induced OSAHS-associated PHT. A previous study has identified that many different pathogeneses, including hepatocellular carcinoma, cervical cancer, and ovarian cancer, were caused by miR-130a, and many genes which have a strong relationship with different cancer pathways have been identified and validated as targeted genes of miR-130a, such as the *GAX* gene.^[19]^ Meanwhile, another study assumed that the expression of *GAX* gene is more or less regulated by miRNAs and confirmed that the *GAX* 3′-UTR miR-130a sequences gave serum responsiveness to the psiCHECK2 reporter plasmid and the expression of *GAX* was significantly downregulated by miR-130a in a manner dependent on the presence of its 3′-UTR miR-130a consensus sequences.^[30]^ Bertero et al^[31]^ indicated that given their inherent pleiotropic actions to limit multiple gene targets simultaneously, miRNAs may be regarded as an important factor to provide comprehensive and integrated control of PHT.

Our study showed that the transcriptional activity of *GAX* gene was lower in the miR-130a mimic group than that in the control and minic-NC groups and higher in the miR-130a inhibitor group than that in the control and inhibitor-NC groups. Furthermore, the expression of *GAX* was decreased in the miR-130a mimic group as compared to the control and minic-NC groups and increased in the miR-130a inhibitor group as compared to the control and inhibitor-NC groups. In the line with our study, Chen and Gorski^[30]^ have identified that miR-130a could affect *GAX* expression and it may play an important role in regulating *GAX* gene activity in endothelial cells (ECs). Besides, it also has been reported that miR-130a has the inhibitory effects both on *GAX* in endothelial cell proliferation, migration, and HoxA5 in tube formation in vitro.^[32]^

Previous evidences also indicated that pathological phenotype modulation of VSMCs plays an important part in the growth of many different types of cardiovascular diseases such as postangioplasty restenosis, atherosclerosis, and hypertension, and *GAX* maintains VSMCs contractile phenotype and monitors VSMCs proliferation and migration by targeting the Rap1A gene.^[24]^ Our study indicated that expressions of ET-1 and VEGF were negatively correlated with the expression of *GAX*, whereas expressions of NO and SOD were positively correlated with *GAX* expression. Evidences had supported that the *GAX* gene may be a transcription factor that as pleiotropic regulator of cell fate, functioning, and regulate cell growth and viability in either a positive or negative way.^[33]^

Lee et al^[34]^ validated that miRNAs have been reported to be main factors of regulating cell apoptosis, proliferation and differentiation. Also, miRNAs are important regulators of gene expression in numerous biological processes and may regulate the gene expression in all major cellular processes, including metabolism and cell cycle.^[35,36]^ Meanwhile, the previous study has suggested that miRNAs have a close relationship with the development and progression of human cancers, including growth, apoptosis, invasion, and metastasis.^[37]^ And our result demonstrated that compared with the control and mimic-NC groups respectively, the miR-130a mimic group showed a raised rate of cell apoptosis. But compared with the control and inhibitor-NC groups, the miR-130a inhibitor group had reduced cell apoptosis rate. Li et al^[38]^ have suggested that over-expression of miR-130a could result apoptosis in A562 cells, which promote the growth inhibitory properties of miR-130a.

In summary, our findings suggest that miR-130a may be involved in the development of OSAHS-associated PHT by down-regulating *GAX* gene. miR-130a could down-regulate the expression of *GAX* and promote tube formation, thereby inducing cell apoptosis of HUVECs and the development of PHT. However, several limitations in the present investigation still existed that merit our further exploration. Due to its little attention paid to such other factors as age and medical history, and less data about the effect of regulation of miR-130a and *GAX* gene on normal cells in our study, which are likely to affect the outcomes, future studies with larger sample size are needed to provide deep investigation about how miR-130a functions on the OSAHS-associated PHT, and more advanced technology will be used to overcome those limitations.

## Acknowledgments

The authors would like to thank all participants enrolled in the present study. They would also like to acknowledge the reviewers for their helpful comments on this paper.
